The article "Early Clinical Outcomes of ACL Reconstruction Using Semitendinosus Tendon Combined with LARS Synthetic" was published in 2022. Journal: Comput Math Methods Med.

# Early Clinical Outcomes of ACL Reconstruction Using Semitendinosus Tendon Combined with LARS Synthetic

**DOI:** 10.1155/2022/2845114

**Published:** 2022-09-30

**Authors:** Baocai Zhang, Peng Xiang, Shuai Bian, Yibo Wang, Yu Wang, Yuzhuo Ma

**Affiliations:** ^1^The First Operating Room, The First Hospital of Jilin University, Changchun City, Jilin Province 130021, China; ^2^Department of Sports Medicine and Arthroscopic Surgery, The First Hospital of Jilin University, Changchun City, Jilin Province 130021, China; ^3^Nursing Platform of Stroke Center, The First Hospital of Jilin University, Changchun City, Jilin Province 130021, China

## Abstract

**Objective:**

To compare the early clinical outcomes of ACL reconstruction using the augmented semitendinosus tendon combined with LARS synthetic material and the autologous hamstring tendons.

**Methods:**

A total of 68 eligible patients with ACL rupture were reconstructed using either 4-strand autologous hamstring tendons, representing the control group, or the LARS synthetic material augmented grafts. The duration of postoperative swelling and recovery exercise was recorded. Lysholm and IKDC scores were used for evaluation of knee joint function. Lachman and pivot shift tests were conducted to evaluate stability.

**Results:**

The scores of the three knee functions in cases of the augmentation group were significantly higher than those of the control group 6 months after surgery (*P* < 0.05). There were no significant differences in Tegner score in the two groups 12 months after surgery (*P* > 0.05). In general, the augmentation group returned to exercise 12 weeks after surgery, while the control group required 30 weeks.

**Conclusions:**

The present study indicates that synthetic material augmentation grafts allow earlier return to exercise and display more satisfactory results compared with the control group.

## 1. Introduction

Anterior cruciate ligament (ACL) is essential for maintaining stability in the knee joint. It has been established that ACL-deficient knees exhibit damage to intra-articular structures such as the meniscus and cartilage, eventually resulting in serious joint degeneration. Arthroscopic ACL reconstruction is the best therapeutic option in young and active population, while the controversy continues over the choice of the graft tissue. In the past, the BPTB autograft has been considered the gold standard in ACL reconstruction because of its osseous fixation mode. Increasingly, the hamstring tendon autografts have been used as an alternative to the BPTB graft due to the reduced donor site morbidity and significantly improved fixation technique and are currently considered as one of the most common grafts. However, regardless the graft type, autograft requires a long time of maturity following implantation, limiting early exercise postoperation, which may negatively affect recovery. Synthetic ligaments for ACL reconstruction have been widely used since the 1980s. The initial enthusiasm about the introduction of synthetic materials stemmed from lack of donor morbidity, abundant supply, and significant strength. The strength of a synthetic material can be applied to share tension during the process of autologous tendon remodeling, protecting potential weak areas and reducing the risk of secondary injury during rehabilitation training, which can help patients return to activity earlier. The aim of the present study was to compare the early outcome of ACL reconstruction using augmentation of semitendinosus tendons with synthetic material versus 4-strand autologous semitendinosus and gracilis tendons (ST/G) to assess the effectiveness of the two groups regarding knee function. Our hypothesis was that postoperative knee stability was better in the augmented group.

## 2. Patients and Methods

### 2.1. Clinical Data

A total of 68 patients with a torn ACL from June 2018 to February 2019 were included in the present study (Table 1). Patients were diagnosed using a pivot shift test and magnetic resonance imaging. Each patient was informed in detail of the nature of their injury and the possible surgical procedures. Each received either an augmented semitendinosus tendon with synthetic material (LARS, L130605B) or 4-strand ST/G, representing the control group, as a graft. The patients were assigned by a single-blind quasirandomization. After passing the inclusion/exclusion criteria and giving consent for the study, they were numbered serially, and alternate numbers were assigned to the two groups. The surgeon was not informed of the group to which a patient was assigned until before surgery. There were 36 cases in the augmentation group, of which 5 cases were complicated by a posterior horn tear of the medial meniscus and 4 with posterior horn tear of the lateral meniscus. There were 32 cases in the control group, of which 4 cases were complicated by posterior horn tear of the medial meniscus and 6 with posterior horn tear of the lateral meniscus. The two groups were comparable in terms of gender, age, period between injury and surgery, and preoperative knee joint function score. All procedures were approved by the local ethical committee and performed by a single senior surgeon. All subjects provided signed informed consent.

### 2.2. Inclusion and Exclusion Criteria

Inclusion criteria: patients suffering their first ACL injury, with no history of knee surgery; professional sports injuries, requiring surgery to continue a sports career; pursuing high quality of life, hoping to return to exercise quickly.

Exclusion criteria: patients with complicated medial or lateral collateral ligament injury, complicated posterior cruciate ligament injury, complicated joint cartilage injury requiring microfracture or osteochondral transplantation, ACL reconstruction adopting an alternative fixation method were excluded. Patients with incomplete clinical information or cognitive impairment and mental abnormalities were also excluded.

### 2.3. Surgical Technique

#### 2.3.1. Graft Preparation of the Augmentation Group

The semitendinosus tendon of the affected limb was excised using conventional methods. LARS synthetic material of an appropriate length and width and a single semitendinosus tendon were laminated and woven together and then folded into two strands, with synthetic material completely wrapping around the semitendinosus tendon, the two edges closed with high-strength sutures to complete preparation of the graft, which had a diameter of 8 mm, and so was the control group. The graft was then soaked in vancomycin saline solution for 10 minutes (Figure 1).

#### 2.3.2. Arthroscopic Graft Installation

Arthroscopic examination was performed using standard anteromedial and anterolateral approaches. Any remaining ACL with synovial covering was preserved as far as possible. All patients underwent arthroscopic single bundle ACL reconstruction. An appropriate femoral offset guide was placed at a 2 or 10 o'clock position for the left or right knees to cover the footprint zone of the anteromedial bundle. The tibial tunnel was positioned as forward as possible, to ensure it did not conflict with the intercondylar fossa. The femoral end of the graft was suspended and fixed with a tight cord (Arthrex, 3.5 mm), while the tibial end was fixed with a bioresorbable screw (Arthrex, 8 mm) combined with an anchor (Arthrex, SwiveLock, 4.75 mm).

### 2.4. Postoperative Rehabilitation

#### 2.4.1. Augmentation Group

Isometric contraction of the quadriceps femoris and ankle pump exercises were conducted immediately following recovery from anesthesia. Knee flexion increased gradually to complete flexion and extension and full weight bearing using a brace within the first 2 weeks. Cycling and jogging were permitted 4 weeks postoperatively. Return to full exercise occurred 3 months after surgery.

#### 2.4.2. Control Group

Isometric contraction of the quadriceps femoris and ankle pump exercise were conducted immediately following recovery from anesthesia. Knees were bent to 90 degrees, and partial weight bearing was permitted using crutches during the first week. Static stepping for balance was allowed for 2 weeks followed by full weight bearing after 4 weeks postoperatively, and cycling and swimming 3 months postoperatively. A gradual return to exercise occurred 6-9 months after surgery.

### 2.5. Follow-Up and Evaluation

All cases were followed up for at least 12 months in strict accordance with the advice from a clinician. The duration of postoperative knee joint swelling evaluated by floating patella test, the duration of the period before return to exercise, and complications such as joint stiffness, infection, and retear were recorded for each patient. The Lysholm score [1], Tegner activity score [2], and IKDC scores [3] were recorded on 4 occasions: preoperatively and after 3, 6, and 12 months. At the final follow-up examination, Lachman and pivot shift tests were conducted for knee stability evaluation.

### 2.6. Statistical Analysis

Prism 6 (GraphPad) statistical software was used to analyze patient data. Measurement data are expressed as means ± SDs and functional score values recorded during follow-up examinations analyzed statistically using a one-way ANOVA and observation results by *t*-tests. A chi-square test was used to compare count data. Differences in which *P* < 0.05 were considered statistically significant.

## 3. Results

### 3.1. Postsurgical Follow-Up

All patients completed a successful follow-up plan. The mean duration of postoperative swelling was 8 days (range: 3-22 days) in the augmentation group and 14 days (range: 10-30 days) in the control group. The augmentation group began to return to exercise 12 weeks (range: 8-20 weeks) after surgery, while the control group was fully exercising 20 weeks (range: 24-40 weeks) after surgery. No patients experienced subjective instability of the knee joint. Objective examination (Table 2) indicated that stability of the knee joint within the augmentation group was greater than that of the control group one year after surgery. At the final follow-up examination, 2 cases underwent arthroscopic secondary exploration for removal of tibial screws (Figure 2).

### 3.2. Knee Joint Functional Score

#### 3.2.1. Comparative Analysis between Groups

There was no significant difference in three knee joint functional scores between the two groups preoperatively (*P* > 0.05). All scores in the augmentation group were significantly higher than those in the control group 3 and 6 months postoperatively (*P* < 0.05). There was no significant difference in Tegner score between the two groups 12 months after surgery (*P* > 0.05), while the Lysholm and IKDC scores in the augmentation group were 97.9 ± 1.9 and 96.9 ± 2.5, respectively, higher than the scores in the control group, at 94.6 ± 1.7 and 93.7 ± 2.1, respectively (*P* < 0.05), although the differences were substantially smaller than at earlier time points. This demonstrates that differences in functional scores in the two groups gradually narrowed as recovery time progressed, being closest at 12 months postoperatively.

#### 3.2.2. Comparative Analysis Intragroup

The increase in the three knee joint functional scores in the augmentation group was the largest in the first 3 months after surgery and lower in the second 3 months, while being the lowest from 6 to 12 months postoperatively. Conversely, in the control group, the increase in knee joint functional scores was the smallest in the first 3 months, while the largest in the period from 6 to 12 months postoperatively (Figures 3–5).

### 3.3. Postoperative Complications

There were 2 cases suffering knee crepitus, following surgery in the augmentation group and 6 cases in the control group. One patient in the augmentation group developed fever after surgery. The infection was eliminated and bacterial culture of the joint fluid was negative. In the control group, 2 cases still had limitations in bending of their knees 3 months after surgery, which were improved by manipulation during outpatient visits. No complications were observed, such as screw loosening, infection, reactive synovitis, bone tunnel enlargement, or retear.

## 4. Discussion

Over recent years, ST/G has become a common autologous grafting procedure for reconstruction of the ACL. However, postoperative ligament relaxation and retear are not uncommon. Literature reports indicate these are related to gender, age, level of exercise, and graft diameter [4]. A cohort study indicated that for every 0.5 mm increase in graft diameter, postoperative revision rate decreased by 14% [5]. Park et al. [6] followed up 296 patients with ST/G ACL reconstruction and found that recovery of knee joint function in grafts with a diameter greater than or equal to 8 mm was significantly greater than that smaller than 8 mm. However, the diameter of an autologous graft is related to the patient's native tendon, which surgeons cannot control. Autologous tendons undergo necrosis, revascularization, and replacement of collagen fibers and finally become shaped and reconstructed into a substitute ligament close to the biological characteristics of an ACL following implantation, its strength correspondingly changing from strong to weak and then gradually increasing. The process lasts for 6 to 9 months or even longer [7, 8]. The high risk of ligament laxity during this period limits the recovery of early activity. Aboalata et al. [9] believed that grafts augmented by high strength sutures could reduce the ligament laxity ratio in patients with a high body mass index and narrow graft (diameter 7 or 7.5 mm).

Synthetic ligaments, in which no revascularization process is required, can exert large mechanical effects immediately following implantation. However, they cannot achieve the biomechanical characteristics of ACL due to the lack of viscoelasticity and occurrence of abrasion [10]. The combination of a synthetic ligament and autogenous tendon can ensure sufficient thickness and length of the graft, and the use of high-strength artificial materials to maintain the initial stability of the joint can protect an autogenous tendon so that the creep period is endured uneventfully, ensuring that early postoperative functional exercise can be safely undertaken, while autogenous tendons can compensate for the deficiency of fatigue decay of the synthetic materials following remodeling. In the present study, standard 4-strand ST/G reconstruction was used as a control, and functional recovery of the knee following augmented reconstruction was evaluated in terms of the subjective assessment of patients, evaluation of clinicians and objective motor capability. The results indicate that the patients in the augmentation group began to return to exercise 12 weeks after surgery, significantly earlier than the 30 weeks in the control group. The three knee joint scores of patients in the augmented group were higher than those in the control group 3 and 6 months after surgery, indicating that knee joint function had recovered more quickly. The Tegner score in particular, which reflects motor capability, improved most significantly 3 months after surgery but was not significantly different in either group after 12 months, indicating that the advantage of this technique is functional improvement during the early stages of recovery.

As early as the 1980s, Kennedy et al. [11] first proposed a ligament augmentation device (LAD), used mainly for *in situ* repair of partial ACL laceration. Kdolsky et al. [12] utilized the Kennedy-LAD technique to treat 66 patients with ACL laceration and followed up for 5-8 years, finding that 75% of the patients recovered preinjury levels of movement following surgery. Nakayama et al. [13] reported that 92% of 50 athletes returned to sporting activities one year after ACL reconstructive surgery using Leeds-Keio augmented autologous ligaments. However, due to limitations in the development of materials science, many negative reports have been published.

With the extensive use of LARS ligament products in France, good therapeutic effects have been achieved. Some researchers [14] have recommended the use of a hollow LARS ligament combined with autologous tendon for ACL reconstruction in patients with poor donor ligament quality, but this method uses only a simple overlap of synthetic material of the two types of graft, which is entirely exposed in the joint cavity and with the same risk of complications as the standard LARS ligament. The maximum load for strips of LARS synthetic material selected in the present study was 3600 N, satisfying the requirements of the mechanical strength of an ACL (1730 ± 270 N). Postoperative nuclear magnetic resonance imaging clearly displayed the structure of the graft, completely wrapped around an autologous tendon (Figure 6), which was able to exert mechanical effects while avoiding the inherent complications of the synthetic material, the incidence of ligament relaxation significantly lower than that of the control group assessed during the one-year follow-up examination. In addition, we used suspension fixation technology, which did not require strict use of absolutely equal graft lengths during surgery, providing excellent fault tolerance compared with conventional LARS reconstruction.

Although removal of any remaining ACL assists in locating the intra-articular bone tunnel and improves the accuracy of surgical procedure, histological studies have confirmed that an abundant blood supply and proprioceptors are present in ligaments and the synovium [15]. In the present study, all patients underwent reconstruction with remnant preservation [16]. The remnant ACL was as far as possible pulled into the bone tunnel or tunnel portal when the graft was installed. The synovium attached to the edge of femoral intercondylar fossa was retained to promote recovery of proprioception following surgery. In addition, only the semitendinosus tendon was excised in the augmentation group, preserving the function of the gracilis muscle.

The sample size of this study was limited and the duration of follow-up not extensive. The clinical value of the study is to some degree compromised, and in the future, a larger sample size and longer duration of follow-up observation are required.

## 5. Conclusions

Compared with standard 4-strand ST/G, LARS synthetic material augmentation of the semitendinosus tendon for ACL reconstruction was able to achieve greater knee joint stability and more satisfactory results, especially in patients who require early recovery of high-level exercise.

## Figures and Tables

**Figure 1:** The preparation process of augmented graft: (a) graft was woven; (b) the reverse side; (c) final appearance of the augmented graft.

**Figure 2:** Magnified observation: augmented graft with synovial sheath and infiltrating vessels during the 12-month follow-up examination.

**Figure 3:** Lysholm scoring of the two groups was compared pre- and postoperatively (∗ stands for *P* < 0.05, ∗∗ stands for *P* < 0.01, and ∗∗∗ stands for *P* < 0.001, ns = not significant).

**Figure 4:** 4IKDC scoring of the two groups was compared pre- and postoperatively (∗ stands for *P* < 0.05, ∗∗ stands for *P* < 0.01, and ∗∗∗ stands for *P* < 0.001, ns = not significant).

**Figure 5:** Tegner scoring of the two groups were compared pre- and postoperatively (∗ stands for *P* < 0.05, ∗∗ stands for *P* < 0.01, and ∗∗∗ stands for *P* < 0.001, ns = not significant).

**Figure 6:** MRI evaluation following ACL reconstruction using an augmented graft. Sagittal view: normal shape of the graft in the joint and synthetic material wrapped around the autogenous tendon. Coronal view: femoral tunnel is completely filled with the graft.

**Table 1:** Demographics of the augmented and control groups.

Group	M/FM	Age	Time to surgery	Lysholm score	Tegner score	IKDC score
Enhance	30/6	27 (17-37)	2.2 (1-6)	46.7 ± 3.4	2.1 ± 0.6	49.2 ± 3.8
Control	24/8	33 (21-42)	3.6 (1-8)	45.1 ± 3.0	2.1 ± 0.5	47.5 ± 3.5

**Table 2:** Lachman and pivot shift test 12 months after surgery.

Group	Lachman			Pivot shift		
	0	1+	2+	0	I	II
Enhance (*n* = 36)	34	2	0	36	0	0
Control (*n* = 32)	26	4	2	29	3	0

## Data Availability

The datasets used and analyzed during the current study are available from the corresponding author upon reasonable request.
